RETRACTED

# The Candida albicans Exocyst Subunit Sec6 Contributes to Cell Wall Integrity and Is a Determinant of Hyphal Branching

**DOI:** 10.1128/EC.00028-15

**Published:** 2015-06-29

**Authors:** Alba A. Chavez-Dozal, Stella M. Bernardo, Hallie S. Rane, Gloria Herrera, Vibhati Kulkarny, Jeanette Wagener, Iain Cunningham, Alexandra C. Brand, Neil A. R. Gow, Samuel A. Lee

**Affiliations:** a Section of Infectious Diseases, New Mexico VA Healthcare System, Albuquerque, New Mexico, USA; b Division of Infectious Diseases, University of New Mexico Health Science Center, Albuquerque, New Mexico, USA; c School of Medical Sciences, Institute of Medical Sciences, University of Aberdeen, Aberdeen, United Kingdom

## Abstract

The yeast exocyst is a multiprotein complex comprised of eight subunits (Sec3, Sec5, Sec6, Sec8, Sec10, Sec15, Exo70, and Exo84) which orchestrates trafficking of exocytic vesicles to specific docking sites on the plasma membrane during polarized secretion. To study *SEC6* function in Candida albicans, we generated a conditional mutant strain in which *SEC6* was placed under the control of a tetracycline-regulated promoter. In the repressed state, the tetR-*SEC6* mutant strain (denoted tSEC6) was viable for up to 27 h; thus, all phenotypic analyses were performed at 24 h or earlier. Strain tSEC6 under repressing conditions had readily apparent defects in cytokinesis and endocytosis and accumulated both post-Golgi apparatus secretory vesicles and structures suggestive of late endosomes. Strain tSEC6 was markedly defective in secretion of aspartyl proteases and lipases as well as filamentation under repressing conditions. Lack of *SEC6* expression resulted in markedly reduced lateral hyphal branching, which requires the establishment of a new axis of polarized secretion. Aberrant localization of chitin at the septum and increased resistance to zymolyase activity were observed, suggesting that C. albicans Sec6 plays an important role in mediating trafficking and delivery of cell wall components. The tSEC6 mutant was also markedly defective in macrophage killing, indicating a role of *SEC6* in C. albicans virulence. Taken together, these studies indicate that the late secretory protein Sec6 is required for polarized secretion, hyphal morphogenesis, and the pathogenesis of C. albicans.

## INTRODUCTION

Exocytosis is an important process that plays a fundamental role in polarized growth in fungi. Exocytosis occurs when cargo-filled vesicles fuse with specific domains of the plasma membrane to provide material needed for cell wall synthesis and expansion. The final stages of polarized growth have been extensively studied in the model yeast Saccharomyces cerevisiae, and they require a highly conserved structure known as the exocyst complex (1, 2). This complex is composed of eight subunits, Sec3, Sec5, Sec6, Sec8, Sec10, Sec15, Exo70, and Exo84 (2), which function in providing spatiotemporal information for the recruitment and tethering of secretory vesicles. The process culminates when vesicles are delivered and tethered to the target membrane via SNARE-mediated membrane fusion, thereby completing the final steps of exocytosis. We have undertaken a detailed pathogenesis study in the role of the late stages of secretion; our work involves the detailed study of the components of the exocyst and SNARE complexes. We previously showed that the Candida albicans t-SNARE proteins Sso2 and Sec9 are required for hyphal growth and secretion (3). Here, we present our findings of the role of the exocyst subunit Sec6 in C. albicans secretion and filamentation.

RETRACTED

In S. cerevisiae, S*EC6* was originally discovered as a temperature-sensitive secretion mutation (4–6). *SEC6* is essential for viability in S. cerevisiae, and a number of conditional mutant phenotypes associated with defective Sec6 function have been described. For example, accumulation of membrane-enclosed 80- to 100-nm vesicles and abnormal endomembrane morphology occur when a *SEC6* conditional mutant strain (S. cerevisiae *sec6-4*) is grown at the restrictive temperature (5). Further, when grown at the permissive temperature, both wild-type Sec6 and Sec6-4 proteins localize to buds and septa; however, when these strains are grown at restrictive temperature, Sec6-4, but not wild-type Sec6, is mislocalized (6). This temperature-sensitive strain is also defective in invertase secretion (4) and polarized growth (7). The exocyst complex forms in the *sec6-4* mutant at the restrictive temperature, but vesicle accumulation is still observed in the cytoplasm (8). In addition, S. cerevisiae Sec6 interacts with the plasma membrane t-SNARE Sec9, suggesting that the Sec6-Sec9 interaction is a critical intermediate in the assembly of SNARE complexes (8). Several studies have also suggested that the protein Sec1 interacts with Sec6 to regulate SNARE complex assembly (9, 10). It is thought that Sec6 interacts with the exocyst after Sec6 releases Sec9, and Sec1 is recruited simultaneously for coordinated SNARE complex formation and membrane fusion (10).

*SEC6* function has been studied in multiple model systems, including Drosophila melanogaster (11), Caenorhabditis elegans (12), and S. cerevisiae (4–10), but there are no reports of its role in trafficking and polarized secretion in the pathogenic yeast Candida albicans, which has a more complex life cycle than S. cerevisiae, as it requires polarized secretion to be differentially regulated during growth in the yeast or hyphal stage. C. albicans is a polymorphic fungus of significant medical importance (13, 14) and has been used as a model for studying the molecular mechanisms of fungal pathogenesis, including polarity, secretion, and filamentation (15–17). Previous studies of the late secretory pathway in C. albicans (for example, the study of Sec3, Sec2, and the t-SNARE proteins Sso2 and Sec9) provided evidence for a key role of the exocyst and SNARE proteins in vesicle-mediated secretion and polarized hyphal growth of C. albicans (3, 18, 19). Therefore, we generated a C. albicans tetracycline-regulated *SEC6* mutant strain to further investigate the role of the exocyst in polarized secretion and filamentation. We found that C. albicans Sec6 plays multiple roles in vegetative growth, cell wall biosynthesis, and virulence of this fungus.

RETRACTED

## MATERIALS AND METHODS

### Strains and media.

All strains used in this study are listed in Table 1. The *URA3*-complemented wild-type strain, THE1-CIp10 (20), was used as a control for all the experiments performed. Strains were grown at 30°C in YPD (1% [wt/vol] yeast extract, 2% [wt/vol] peptone, 2% [wt/vol] glucose) or CSM (complete synthetic medium; 0.67% [wt/vol] yeast nitrogen base without amino acids, 2% [wt/vol] glucose, 0.079% [wt/vol] complete synthetic mixture), supplemented with uridine (80 μg/ml) where required. Uracil auxotrophs were selected on 5-fluoroorotic acid (FOA) medium (CSM supplemented with 0.1 mg/ml uridine and 0.7 mg/ml FOA). Doxycycline (DOX) was added to a final concentration of 20 μg/ml to repress expression of *SEC6*. Solid media were prepared by adding 2% (wt/vol) agar.

**TABLE 1:** Candida albicans strains used in this study

Strain name	Parent	Genotype	Source
THE1	CAI8	*ade2*::*hisG*/*ade2*::*hisG ura3*::*imm434*/*ura3*::*imm434 ENO1*/*eno1*::*ENO1-tetR-ScHAP4AD-3×HA-ADE2 SEC6*/*SEC6*	22
THE1-CIp10	THE1	*ade2*::*hisG*/*ade2*::*hisG ura3*::*imm434*/*ura3*::*imm434 ENO1*/*eno1*::*ENO1-tetR-ScHAP4AD-3×HA-ADE2 RPS1/RPS1*::*URA3 SEC6*/*SEC6*	20
*sec6*Δ/+	THE1	*ade2*::*hisG*/*ade2*::*hisG ura3*::*imm434*/*ura3*::*imm434 ENO1*/*eno1*::*ENO1-tetR-ScHAP4AD-3×HA-ADE2 SEC6*/*sec6*Δ::*dpl200-URA3-dpl200*	This study
*sec6*Δ/+ FOA	*sec6*Δ/+	*ade2*::*hisG*/*ade2*::*hisG ura3*::*imm434*/*ura3*::*imm434 ENO1*/*eno1*::*ENO1-tetR-ScHAP4AD-3×HA-ADE2 SEC6*/*sec6*Δ::*dpl200*	This study
tetR-*SEC6*	*sec6*Δ/+ FOA	*ade2*::*hisG*/*ade2*::*hisG ura3*::*imm434*/*ura3*::*imm434 ENO1*/*eno1*::*ENO1-tetR-ScHAP4AD-3×HA-ADE2 URA3*-tetR-*SEC6*/*sec6*Δ::*dpl200*	This study
T-CDC10gfp	THE1-CIp10	*ade2*::*hisG/ade2*::*hisG ura3*::*imm434/ura3*::*imm434 ENO1/eno1*::*ENO1-tetR-ScHAP4AD-3×HA-ADE2 RPS1/RPS1*::*URA3 SEC6/SEC6 CDC10/CDC10-GFP*::*NAT1*	This study
tSEC6-CDC10gfp	tetR-*SEC6*	*ade2*::*hisG/ade2*::*hisG ura3*::*imm434/ura3*::*imm434 ENO1/eno1*::*ENO1-tetR-ScHAP4AD-3×HA-ADE2 URA3*-tetR-*SEC6/sec6*Δ::*dpl200 CDC10/CDC10-GFP*::*NAT1*	This study

RETRACTED

### Preparation of plasmid and genomic DNA.

Plasmids were maintained in Escherichia coli DH5α cells (Invitrogen, Carlsbad, CA) grown in LB medium (1% [wt/vol] tryptone, 0.5% [wt/vol] glucose, and 1% [wt/vol] NaCl) with ampicillin (100 μg/ml) at 37°C. Plasmid DNA was prepared from E. coli strains by using the PureYield plasmid miniprep system (Promega, Madison, WI). Genomic DNA was extracted from yeast cells by using the MasterPure yeast DNA purification kit (Epicentre Biotechnologies, Madison, WI) according to the manufacturer's instructions, with the addition of a 1-h incubation step on ice after the addition of the protein precipitation reagent.

### Construction of a tetracycline-regulated C. albicans *SEC6* mutant strain.

Table 2 lists the primers used in this study. Strain construction was performed as follows. First, we deleted one allele of *SEC6* in the THE1 background to generate the strain *sec6*Δ/+ via a PCR-based gene disruption strategy previously described by Wilson et al. (21), using primers SEC6-5DR and SEC6-3DR and plasmid pDDB57 as a template. Colonies were verified by allele-specific PCR using primers SEC6-5Det and SEC6-3Det, which anneal to regions up- and downstream of the *SEC6* open reading frame, respectively. Colonies that contained the correct integration of the *URA3* disruption cassette (*dpl200*::*URA3*::*dpl200*) were designated *sec6*Δ/+. To regenerate uracil auxotrophy, the *sec6*Δ/+ strains were plated on agar medium containing 5-FOA to induce loss of *URA3* by *cis*-recombination between the flanking *dpl200* repeats. The resultant 5-FOA-resistant colonies were screened via PCR for the *SEC6*/*sec6*Δ::*dpl200* genotype by using primers SEC6-5Det and SEC6-3Det. Next, the *tetO* promoter from plasmid p99CAU1 (22) was inserted upstream of the remaining *SEC6* allele in the *sec6*Δ/+ FOA strains by using the PCR-based strategy previously described by Bates et al. (23) and primers tetSEC6-5DR and tetSEC6-3DR. Transformants were screened using primers tetSEC6-5Det and tetSEC6-3Det; the final constructed strain was named tetR-*SEC6* (denoted as tSEC6 in the manuscript). Strain construction was verified by Southern blotting. In brief, genomic DNA digested with HindIII and EcoRV was separated on a 0.8% (wt/vol) agarose gel. DNA fragments were transferred to a positively charged nylon membrane (Roche Applied Science, Indianapolis, IN). A digoxigenin (DIG)-labeled probe (nucleotide [nt] −500 to nt 500 of orf19.5463) was prepared from genomic DNA isolated from strain THE1 with primers SEC6-5Sblt and SEC6-3Sblt (Table 2) and reagents supplied in the PCR DIG probe synthesis kit (Roche Applied Science, Indianapolis, IN). Detection of HindIII and EcoRV DNA fragments of the expected sizes for the wild-type allele (*SEC6*; 2.4 kb), *sec6*Δ/+ allele (*sec6*Δ::dpl200-*URA3*-dpl200; 2.1 kb), *sec6*Δ/+ FOA allele (*sec6*Δ::dpl200; 0.8 kb), and tSEC6 allele (*URA3*-tetR-*SEC6*; 2.5 kb and 0.5 kb) confirmed the genotype of each construct (data not shown).

RETRACTED

**TABLE 2:** Primers used in this study

Primer	Primer sequence (5′ → 3′)
SEC6-5DR	CATTAGTATATAGGAAGAGAAAAAAAAAAAAAAATGAACAACAAAAAAAGAATCTCGTTTACTCTCTCCACGTCGTTTTCCCAGTCACGACGTT
SEC6-3DR	CCGGTTGCCAAACGCAAGCTTGTCATTCCTACAACTATCAAACTCCCTAAAAAACCTAGACTTGCCCGCCTGTGGAATTGTGAGCGGATA
TetSEC6-5DR	CAACCCGTATGGTAGAAGGTACACGAAAAAACATTAGTATATAGGAAGAGAAAAAAAAAAAAAAATGAACGTAATACGACTCACTATAGGG
TetSEC6-3DR	TGCCTATCTTGGCCAAATCATCTTCCAATTTGATCAATTCACTGATCTTAGATAACGTTGAATCGCTCATCTAGTTTTCTGAGATAAAGCTG
SEC6-5Det	CCGCCGCAAGGGTTTGTGCC
SEC6-3Det	TCTGGGCATGGAAAATCTCG
tetSEC6-5Det	GGGGTGAACAAAGTGCCAAC
tetSEC6-3Det	CGCAGGTGCAGATTGATTCG
RT-SEC6-5Det	GAATGCGCCGGACATTTACC
RT-SEC6-3Det	ACTTTTTGGTGGCCTGTGGA
SEC6-5Sblt	GGCAGCAGACTTTTTTGGGG
SEC6-3Sblt	AAATCGTCCGACAACCTCGT
CDC10-GFP/NAT1-5DR	TTTGAAGAACGCCTCTGGTGTGCCAAATGCTCCTATGTTCCAATCAACTACAGGTACTGCTGCTGCTAGAGGTGGTGGTTCTAAAGGTGAAGAATTATT
CDC10-GFP/NAT1-3DR	AACACACAAAAGAAGAGGAATACAAAAAAGTAAAATCACATTATATCAATAACAAACATTATTTATCTATCGTTAGTATCGAATCGACAGC
CDC10-5Det	CAAAAAGATCAAGGGCAAAC
CDC10-3Det	ATAAAATCTCGAGTGGGAAA

### Analysis of *SEC6* gene expression.

Expression of *SEC6* in the THE1-CIp10 control strain and tSEC6 after 2 and 4 h of growth in medium (with or without DOX) was assayed using reverse transcriptase PCR (RT-PCR) (see Fig. S1 in the supplemental material). Cells from an overnight culture were resuspended in fresh YPD with or without DOX and grown for 2 or 4 h. RNA was isolated using the RiboPure yeast RNA isolation kit (Life Technologies, Grand Island, NY) according to the manufacturer's instructions. RT-PCR was performed using the Access RT-PCR system (Promega, Madison, WI) according to the manufacturer's protocol, using primers RT-SEC6-5Det and RT-SEC6-3Det (Table 2) and 1 μg total RNA as the template. The absence of contaminating DNA was tested in parallel PCR-based analyses.

### Analysis of *in vitro* growth.

*In vitro* growth was assessed using liquid and solid media. Growth on solid medium was carried out by spotting serial dilutions of cells on CSM with or without DOX, with cells prepared as described previously (24). Plates were incubated at 30°C for 24 h. Growth in liquid medium was assessed at two different temperatures (30 and 37°C) by measuring the optical density at 600 nm (OD_600_) at fixed intervals via an Ultraspec 2100 Pro spectrophotometer (GE Healthcare Life Sciences, Piscataway, NJ), after cells from overnight cultures were washed and transferred to fresh CSM with or without DOX and diluted to a starting OD_600_ of 0.1. Optical densities were recorded, and growth curves were generated using GraphPad Prism 6 (GraphPad Software, Inc., La Jolla, CA). At each time point, cells were counted using a hemocytometer, and approximately 300 cells were plated onto YPD agar to determine viability by counting CFU. CFU determinations were performed in triplicate independently.

RETRACTED

### Assessment of cellular and vacuolar morphologies.

Strains THE1-CIp10 and tSEC6 were grown overnight in 5 ml YPD, resuspended to an OD_600_ of 0.1, and incubated for 24 h in the presence or absence of DOX. Cells were visualized via differential interference contrast (DIC) microscopy (Carl Zeiss AG, Jena, Germany). To simultaneously stain vacuoles with FM4-64 [*N*-(3-triethylammoniumpropyl)-4-(6-(4-(diethylamino) phenyl) hexatrienyl) pyridinium dibromide] and CMAC (7-amino-4-chloromethyl coumarin) (both from Life Technologies, Grand Island, NY), cells were grown for 20 h in the presence or absence of DOX. Cells were inoculated into fresh medium and grown to early log phase (total incubation time, 24 h). For FM4-64 staining, cells were resuspended to an OD_600_ of 2 to 4 in YPD with 40 μM FM4-64 and incubated for 15 min at 30°C, resuspended in fresh YPD, and incubated for 45 min at 30°C. After incubation, the cells were resuspended to an OD_600_ of 0.1 in 10 mM HEPES, 5% (wt/vol) glucose, pH 7.4. CMAC was then added to a concentration of 100 μM, and cells were incubated at room temperature for 15 min prior to imaging via epifluorescence microscopy using Texas Red (FM4-64) and DAPI (CMAC) filters (25). Images were acquired and processed using AxioVision 4.7 (Carl Zeiss AG, Jena, Germany). Samples for thin section electron microscopy were prepared as described previously (3) from tSEC6 grown in the presence and absence of DOX for 24 h at 30°C, and micrographs were acquired using a Hitachi H7500 transmission electron microscope (Hitachi High-Technologies Corp., Japan).

### Morphological characterization and counting of bud scars.

Strains THE1-CIp10 and tSEC6 were grown for 24 h in the presence or absence of DOX. Bud scars were visualized by chitin staining in growth medium containing 2 μg/ml calcofluor white (CW; Sigma-Aldrich, St. Louis, MO) for 15 to 30 min. Bud scar patterns were scored as follows: cells with three to five bud scars were considered “axial” if all bud scars were in a single chain, “bipolar” if at least two bud scars were at opposite ends of a cell, and “random” if the pattern was neither bipolar nor axial (26). Cells were visualized using DIC and fluorescence microscopy using a DAPI filter, and image assembly was completed using AxioVision 4.7 (Carl Zeiss AG, Jena, Germany).

RETRACTED

### Sensitivity to cell wall-perturbing agents.

The ability of strain tSEC6 to grow on medium containing cell wall stressors was tested on agar plates in the presence or absence of DOX and compared to that of controls. Plates included CSM with (i) 0.025 μg/ml caspofungin (CAS), (ii) 200 μg/ml Congo red (CR), (iii) 50 μg/ml CW, or (iv) 0.2% (wt/vol) SDS. Overnight cultures of strains tSEC6 and THE1-CIp10 were diluted for this experiment; a total of five 5-fold dilutions (starting at 10^8^ cells/ml) were prepared in 96-well plates, and cells were stamped onto agar plates by using a multiblot replicator (VP 408H; VP Scientific Inc., San Diego, CA). Plates were incubated at 30°C for 24 h.

To test for defects in cell wall composition, cells were grown overnight with or without DOX and treated with Zymolyase 100T (β-1,3-glucanase; Sunrise Products Inc., Waterville, MN) as described previously (27). In brief, exponentially growing cells were adjusted to OD_600_ of 0.5 in 10 mM Tris-HCl (pH 7.5) containing 25 μg/ml of Zymolyase 100T; the decrease in optical density was monitored over 140 min, and light microscopy images were obtained every 20 min (27). Additionally, the number of cells that were unaffected by the zymolyase treatment was determined by counting the number of intact cells over 10 fields per slide per treatment at the time points indicated.

Determination of sensitivity to chitinase was analyzed as described previously (28). Chitinase from Streptomyces griseus (Sigma-Aldrich, St. Louis, MO) was dissolved in 200 mM potassium phosphate buffer (pH 6.0) at 25°C with 2 mM calcium chloride to a final concentration of 1 U/ml of chitinase. Exponentially growing cells were adjusted to an OD_600_ of 0.5 in phosphate buffer containing chitinase and incubated for 2 h. The decrease in optical density was then recorded every 15 min for a total of 2 h.

### Analysis of cell wall composition.

Cell walls from strains THE1-CIp10 and tSEC6 (grown in the presence of absence of DOX) were extracted as previously described (29). In brief, overnight strains were subcultured and grown (with or without DOX, for 24 h at 28°C, with shaking at 250 rpm). Cells were collected (3,000 × *g* for 5 min) and resuspended in deionized water. Cells were fractured in a FastPrep machine (Qbiogene, Carlsbad, CA) using beads for cell disruption. Cell debris was washed five times with 1 M NaCl and resuspended in buffer (500 mM Tris-HCl [pH 7.5], 2% [wt/vol] SDS, 0.3 M β-mercaptoethanol, 1 mM EDTA), boiled for 10 min, and then freeze-dried. For quantification of cell wall components (glucan, mannan, and chitin), 2 M trifluoroacetic acid was used to acid hydrolyze cell walls. Acid was evaporated at 65°C, and samples were washed and resuspended in deionized water. The hydrolyzed cell wall composition was analyzed by high-performance anion-exchange chromatography with pulsed amperometric detection (HPAEC-PAD) in a carbohydrate analyzer system from Dionex (Surrey, United Kingdom). The total concentration of each component was determined by calibration from the standard curves of glucosamine, glucose, and mannose monomers and is reported as a percentage relative to results for the total cell wall.

RETRACTED

### Assay for secreted aspartyl proteases.

Liquid assays for secreted aspartyl proteases were performed as follows: cells from 5-ml overnight cultures were resuspended in 30 ml bovine serum albumin (BSA) medium (0.34% [wt/vol] YNB without amino acids and without ammonium sulfate, 2% [wt/vol] glucose, 0.1% [wt/vol] BSA) to induce production of Sap2 proteases, and the mixtures were incubated for 24 h. Spent medium was removed, and the cells were resuspended to an OD_600_ of 30 in fresh BSA medium containing only 0.01% (wt/vol) BSA. The cell suspension was divided equally, and DOX was added to one sample. Cultures were incubated at 30°C for 24 h with shaking at 250 rpm. Cell-free culture supernatant was used for SDS-PAGE analyses as described previously (20). The triple deletion mutant *sap*Δ(1-3) was included as a control (30). Bands of intact BSA indicate reduced secretion of Saps.

### Assay for lipase secretion.

The assay performed for secreted lipases was a modification of the turbidimetric esterase assay developed by von Tigerstrom and Stelmaschuk (31). Secretion of lipase was induced by growing cells from a standard overnight culture (diluted 1:100) in Tween 80 medium (0.54% [wt/vol] YNB without amino acids, 2.5% [vol/vol] Tween 80). Following incubation at 37°C for 24 h with shaking at 250 rpm, cells were washed twice in 1× phosphate-buffered saline (PBS), concentrated to an OD_600_ of 10 in Tween 80 medium, and incubated for 24 h with or without DOX at 37°C with shaking at 250 rpm. Supernatants from the cultures were tested for secreted lipases in a kinetic assay: 500 μl of cell-free supernatant was added to 5 ml of Tween 20 substrate (2% [vol/vol] Tween 20 in 20 mM Tris-HCl [pH 8.0] and 120 mM CaCl_2_) and incubated at 37°C with shaking at 250 rpm; OD_500_ readings were taken every 15 min for up to 75 min. Tween 20 substrate without lipase was similarly treated and used as a control to correct for background absorbance of the substrate at each time point. The kinetic profiles of the secreted lipases under each growth condition were visualized and compared by plotting the OD_500_ readings over time (31). The turbidimetric assay measures the precipitation of calcium ions by degradation products resulting from lipolytic activity of enzymes secreted into the culture supernatant. The rate of increase in optical density (OD_500_) is proportional to the concentration of lipases present in the supernatant.

RETRACTED

### Filamentation assays.

Filamentation in liquid medium was assayed at 37°C in RPMI 1640 supplemented with l-glutamine (Cellgro, Manassas, VA) and buffered with 165 mM 3-morpholinopropanesulfonic acid (Sigma, St. Louis, MO) to pH 7.0 (“buffered RPMI 1640”). In brief, buffered RPMI 1640 with or without DOX was inoculated with cells from overnight cultures at a final density of 5 × 10^6^ cells/ml, followed by incubation at 37°C with shaking at 200 rpm. Cells were visualized by DIC microscopy after 24 h by using a Zeiss EC Plan-NeoFluar 63×/1.25× oil objective (Carl Zeiss AG, Jena, Germany).

Filamentation was assayed on solid YPD with 10% (vol/vol) fetal calf serum (FCS), Medium 199 supplemented with l-glutamine (M199), and Spider medium, as described previously (24). YPD agar was used for embedded colony observation as described previously (32). All plates were prepared with and without 20 μg/ml doxycycline. Aliquots of 3 μl of cells from overnight cultures were spotted onto agar plates and incubated at 37°C for 24 h. For embedded colony observation, molten YPD agar was cooled to approximately 45°C and cells from overnight cultures were added to a concentration of 20 cells/ml, poured into individual petri dishes, and incubated for 24 h at 30°C. Filamentation was observed with an inverted microscope (Fisher Scientific, Waltham, MA) at 100× and 400× total magnification.

### Determination of hyphal branching patterns.

In order to characterize hyphal branching patterns, strains were grown in YPD with and without DOX for 15 h, and then filamentation was induced at 37°C in liquid YPD plus 20% (vol/vol) FCS (with and without DOX) for 8 h. The numbers of branched and unbranched hyphae were counted and averaged from 100 cells. Bud-shaped or pseudohypha-shaped filaments were discounted. The degree of branching was determined by counting the number of branches emanating from the primary hyphae (33).

### Macrophage killing assays.

The *in vitro* model of macrophage infection with C. albicans was performed as previously published (34). The J774A.1 murine macrophage cell line was purchased from ATCC (American Type Culture Collection, Manassas, VA). Macrophages were grown in high-glucose Dulbecco's modified Eagle's medium (DMEM) supplemented with 10% (vol/vol) FCS at 37°C, 5% CO_2_ for 72 h. Fresh DMEM plus 10% (vol/vol) FCS was inoculated with 2 × 10^5^ macrophages in a final volume of 0.75 ml to seed Lab-Tek chambered slides (Nalge-Nunc, Rochester, NY). Slides were then incubated at 37°C with 5% CO_2_ overnight. Spent medium was removed, and adherent macrophage cells were washed twice with PBS. Overnight cultures of C. albicans strains THE1-CIp10 and tSEC6 were washed three times in PBS and added to DMEM with 10% (vol/vol) FCS, with or without DOX, and 0.75 ml of this cell suspension was used for coincubation with the macrophage cells at a multiplicity of infection of 2. C. albicans cells were coincubated with the adherent macrophage cells overnight at 37°C with 5% CO_2_. Cells were then washed twice with PBS, and macrophage viability was assessed using the LIVE/DEAD viability/cytotoxicity kit (Invitrogen, Carlsbad, CA) following the manufacturer's instructions. Live macrophages from 12 separate fields of each chamber were counted. The experiment was performed independently three times.

RETRACTED

### Visualization of C. albicans septin localization.

To tag with green fluorescent protein (GFP) the septin ring as has been previously described (35), GFP was inserted in frame at the C terminus of *CDC10* by using a nourseothricin selection method (36). Briefly, the *GFP-NAT1* cassette was amplified from plasmid pGFP-NAT1 using primers CDC10-GFP-5DR and CDC10-GFP-3DR; transformation of the cassette into THE1-CIp10 and tSEC6 strains was completed using the lithium acetate method, with a 4-h growth step in YPD added after the heat shock step to allow integration and translation of the *NAT1* gene before exposing the cells to nourseothricin, as described previously (36). Transformants were selected on Difco Sabouraud-dextrose agar (BD, Franklin Lakes, NJ) containing 200 μg/ml nourseothricin (Gold Biotechnology, St. Louis, MO). Primers flanking the *CDC10* open reading frame (Table 2) were used to screen for transformants carrying the *CDC10*-GFP allele. DIC and GFP fluorescence images were acquired after induction of filamentation in buffered RPMI for 6 and 24 h in the presence or absence of DOX and in yeast cells after 24 h in YPD with or without DOX. DIC and GFP fluorescence images were acquired using AxioVision 4.7 software (Carl Zeiss AG, Jena, Germany) and a Zeiss EC Plan-NeoFluar 63×/1.25× oil objective (Carl Zeiss AG, Jena, Germany).

RETRACTED

### Statistical analyses.

Results were analyzed using a one-way analysis of variance and Tukey's multiple comparison test (GraphPad Software, Inc., La Jolla, CA). Results were considered statistically significant if *P* was <0.05 compared to all other treatments.

## RESULTS

### *SEC6* is required for long-term viability in C. albicans.

Since the late secretory gene *SEC6* is essential for viability in S. cerevisiae, we generated a tetracycline-repressible mutant of *SEC6* in C. albicans (denoted strain tSEC6). Expression of *SEC6* in tSEC6 and the control strain, THE1-CIp10, in the absence or presence of DOX was analyzed by RT-PCR (see Fig. S1 in the supplemental material). *SEC6* expression was detected at 2 h in strain tSEC6 in the presence of DOX, but it was not detected after 4 h. Next, we assessed the contribution of *SEC6* to cell growth and viability. No visible difference in growth was observed on solid CSM with or without DOX incubated for 24 h (data not shown). There were no significant differences in OD_600_ values and the rate of growth between the wild-type and mutant strains when grown at either 30°C (Fig. 1A) or 37°C (Fig. 1B), under repressing or derepressing conditions. We also measured cell viability by enumerating CFU at different time points of growth at these temperatures. In the repressed state, tSEC6 cells remained viable for up to 27 and 30 h at 30 and 37°C, respectively (Fig. 1C and D), after which cell death occurred. Based on these observations, all phenotypic assessments were performed at time points that did not exceed a total of 24 h, to ensure that any differences that were observed in tSEC6 with DOX compared to wild-type controls was not a direct result of cell death.

**FIG 1:** *In vitro* growth of the C. albicans tSEC6 mutant strain in the presence or absence of doxycycline. (A) Growth was assessed by measuring OD_600_ values of microcultures at a starting OD_600_ of 0.05 in CSM with or without DOX and incubated with shaking at 30°C. (B) A similar assessment of growth was performed at 37°C. There was no significant difference (*P* > 0.05) in optical density readings after incubation for 34 h. (C) CFU analysis was performed at the indicated time points at 30°C by plating approximately 300 cells from cultures grown in liquid YPD medium and counting CFU (*n* = 3; bars indicate standard deviations [SD]). There was a significant difference (*P* < 0.05) in CFU counts between the tSEC6 mutant strain in the presence of DOX and its controls after 27 h of incubation. (D) Similarly, CFU analysis was performed at 37°C (*n* = 3; bars indicate SD). There was a significant difference (*P* < 0.05) in CFU counts between the tSEC6 mutant strain in the presence of DOX and its controls after 30 h of incubation.

RETRACTED

### Repression of *SEC6* results in altered cell morphology and increased axial bud scar localization.

Wild-type strains have a typical oval-shaped yeast cell morphology (4 to 6 μm in size). In contrast, light and DIC microscopy revealed altered gross cellular morphologies in the tSEC6 strain grown under restrictive conditions. tSEC6 cells were larger than the control strain and formed chain-like structures composed of three to five cells (Fig. 2A). Chains of cells became evident after 8 h under restrictive conditions, when approximately 10% of the cells were enlarged (data not shown); after 24 h, nearly all of the tSEC6 plus DOX cells had this abnormal phenotype (Fig. 2A).

**FIG 2:** Cell morphology of tSEC6 and THE1-CIp10 strains under restrictive and nonrestrictive conditions. (A) Yeast structures were observed after 24 h of incubation in YPD with or without DOX. tSEC6 cells were larger than wild-type yeast cells and formed chains of three to five cells in length. Bar, 10 μm. (B) THE1-CIp10 and tSEC6 were incubated in YPD with or without DOX for 24 h and then stained with calcofluor white, and bud scars were observed under fluorescence microscopy using a DAPI filter. Bud scar position was evaluated by counting 100 cells and classifying the budding pattern. There was a significant increase of axial scar pattern in the tSEC6 with DOX strain and a decrease in bipolar scars (indicated by the asterisks [*P* < 0.001]). Three biological replicates were analyzed. Bars indicate the standard deviations.

We observed an alteration in bud scar distribution in the tSEC6 mutant plus DOX. Bud scar localization can be classified as axial or unipolar (the bud located in the one-third portion closest to the birth scar), bipolar (bud opposite to the birth scar), or random (bud on the middle third of the cell) (26). Wild-type THE1-CIp10 cells displayed a predominantly bipolar bud scar pattern, whereas tSEC6 plus DOX bud scars were predominantly axial (Fig. 2B).

### Repression of *SEC6* results in defective cytokinesis and abnormal septal structure.

The formation of chains of cells suggested that the tSEC6 mutant is defective in cytokinesis. Cytokinesis is the process by which a cell divides its cytoplasm to produce two daughter cells. Cytokinesis is a common process in filamentous fungi and yeast cells, and it is mediated by the formation of septa (37). To determine whether the tSEC6 strain formed normal septa under restrictive conditions, CW was used to stain the chitin of the primary septal plate. Distinct septa were observed in strain THE1-CIp10 with or without DOX and tSEC6 without DOX (Fig. 3A). However, for the tSEC6 strain with DOX, CW staining revealed an increased amount of chitin in the region of the septum (Fig. 3A) similar to that seen in S. cerevisiae strains with mutations in the septins or proteins involved in chitin deposition that localize to the mother-daughter bud neck (37–39). An abnormally thickened septum within a wide bud neck was clearly evident when the tSEC6 mutant was analyzed using thin section electron microscopy (Fig. 3B). The abnormal septal structure and the presence of multiple cellular chains indicated that the absence of *SEC6* produces a defect in cytokinesis.

RETRACTED

**FIG 3:** Bud neck structure and septin localization in strain tSEC6. (A) Strains were incubated for 24 h in YPD with or without DOX, stained with calcofluor white, and observed under a fluorescence microscope using a DAPI filter. Microscopy of cells stained with calcofluor white revealed an increased concentration of chitin at the bud neck in C. albicans tSEC6 strains under restrictive conditions. Bar, 5 μm. (B) Cells were grown in YPD with or without DOX for 24 h and fixed for analysis using thin section electron microscopy. The electron micrographs revealed the presence of a thickened septum in the bud neck of the tSEC6 mutant cultured in the presence of DOX (black arrows). Bar, 2 μm. (C) Strains carrying *CDC10*-GFP alleles were grown in YPD with or without DOX for 24 h. Fluorescence microscopy was used to visualize localization of Cdc10-GFP to sites of polarized growth and septin ring assembly. Strain tSEC6 cultured in the presence of DOX showed septin rings stretched laterally, compared to those found in wild-type control strains. Bar, 5 μm.

The septin Cdc10 localizes to the septin ring that is formed at the bud neck between the mother and daughter cell, marking sites where septum formation occurs. Because the morphology of the septum was abnormal in tSEC6, we asked whether septin localization was altered. Cdc10-GFP was present in the control strains at the mother-daughter bud neck and sometimes appeared as a doublet when cell division had progressed further (Fig. 3C). In contrast, an abnormally elongated septin ring structure was observed in the tSEC6 mutant strain grown under repressing conditions (i.e., with DOX) (Fig. 3C).

### Repression of C. albicans SEC6 expression results in defective endocytosis and accumulation of late endosomes and post-Golgi apparatus secretory vesicles.

The fungal vacuole plays a key role in C. albicans biology and pathogenesis (34). Since defects in vacuolar function result in a number of abnormal pathogenesis-related phenotypes, we visualized the vacuolar integrity by using the fluorescent dyes FM4-64 and CMAC. FM4-64 is a lipophilic dye that binds to cellular membranes and is actively endocytosed to the vacuole, whereas CMAC is a dye that passively accumulates in the vacuolar lumen and inside late endosomes. In addition to its utility as a marker for vacuolar morphology, FM4-64 is also a marker for endocytic trafficking from the plasma membrane to the vacuolar membrane (25). Fluorescence microscopy showed that the control strains (THE1-CIp10 with or without DOX and tSEC6 without DOX) had normal spherical vacuoles, and after 45 min of incubation, FM4-64 was mostly present at the vacuolar membrane (Fig. 4A). In contrast, in the tSEC6 mutant plus DOX, FM4-64 remained primarily at the plasma membrane, indicating an impairment in endocytosis. CMAC staining of the tSEC6 strain plus DOX revealed accumulation of ovoid structures resembling late endosomes, which have been described to be readily visualized with CMAC in Aspergillus nidulans (40). We further investigated the nature of these structures by visualization of tSEC6 under derepressing and repressing conditions using thin section electron microscopy. When grown under derepressing conditions, there was no difference in ultrastructural features of tSEC6 compared to THE1-CIp10 (20). Microscopy images revealed the accumulation of post-Golgi apparatus secretory vesicles (approximate size, 40 to 90 nm) and larger ovoid structures consistent with late endosomes (approximate size, 250 nm) when strain tSEC6 was grown under repressing conditions (Fig. 4B; see also Fig. S2 in the supplemental material).

RETRACTED

**FIG 4:** Accumulation of late endosomes and post-Golgi apparatus secretory vesicles in strain tSEC6. (A) FM4-64 (red membrane stain) and CMAC (blue vacuolar lumen stain) double fluorescent staining was performed to visualize vacuole-related organelles in control and tSEC6 strains grown with or without DOX. Strain tSEC6 growth with DOX accumulated multiple structures which were stained by CMAC. FM4-64 remained at the plasma membrane, in contrast to the controls, where it was actively endocytosed into the vacuolar membrane. Bar, 10 μm. (B) Cells were grown in YPD with or without DOX for 24 h and fixed for analysis using thin section electron microscopy. Representative micrographs are shown: (1) tSEC6 without DOX; (2 to 4) tSEC6 with DOX. The micrographs revealed accumulation of structures resembling post-Golgi apparatus secretory vesicles (black arrows) and late endosomes (white arrows) in the tSEC6 strain grown under repressing conditions that were not present under derepressing conditions. Bar, 500 nm.

### *SEC6* contributes to cell wall integrity.

Our results indicated that chitin content was abnormally increased at the septin ring, suggesting that the chitin/glucan ratio might be altered. To further examine the role of *SEC6* in maintenance of cell wall integrity, we performed a chitinase assay which revealed that strain tSEC6 with DOX had increased resistance to chitinase compared to controls (Fig. 5A). A zymolyase assay to indirectly assess glucan content showed that tSEC6 plus DOX was markedly resistant to zymolyase degradation compared to the control strains (Fig. 5B), suggesting that *SEC6* repression increased the glucan content of the cell wall. Additionally, after zymolyase treatment, we visualized the formation of Candida spheroplasts via light microscopy (Fig. 5C). The number of unaffected cells (after zymolyase treatment) was markedly increased in strain tSEC6 with DOX compared to controls (Fig. 5D). These results are congruent with the turbidity endpoint data observed in the zymolyase kinetic assay.

RETRACTED

**FIG 5:** Qualitative determination of cell wall components via enzymatic assays. (A) Strains were incubated for 24 h with or without DOX, in the presence of chitinase. Chitinase activity was followed spectrophotometrically at a wavelength of 600 nm, at which a decrease in optical density occurs as cell wall material is degraded. Optical density readings were significantly higher for the tSEC6 mutant in the presence of DOX compared to the controls after 2 h of incubation with chitinase, indicating resistance to cell lysis. The asterisk indicates a statistically significant difference (*P* < 0.005) at the time point indicated and later time points. (B) Strains were incubated for 24 h with or without DOX, in the presence of Zymolyase 100T. Zymolyase activity was followed spectrophotometrically at a wavelength of 600 nm. Optical density readings were significantly higher for tSEC6 in the presence of DOX after 45 min of incubation with zymolyase, indicating resistance to cell lysis by zymolyase. The asterisk indicates statistically significant difference (*P* < 0.005) at the time point indicated and later time points. (C) Following incubation with zymolyase, formation of spheroplasts was visualized using light microscopy. Spheroplast formation and cell lysis were reduced in strain tSEC6 grown under restrictive conditions. Bar, 10 μm. (D) The number of cells that were unaffected by zymolyase was determined over time. Three independent experiments were performed in which the number of intact cells over 10 fields per slide per treatment were counted. There was a significant increase in the number of cells that were not affected by zymolyase in strain tSEC6 grown in the presence of DOX as early as at 30 min of incubation with zymolyase compared to the controls. The asterisk indicates a statistically significant difference between wild-type controls and tSEC6 grown with DOX (*P* < 0.005).

RETRACTED

These findings suggested a possible alteration in the content of chitin and glucan in the tSEC6 conditional mutant; therefore, we next assessed growth in the presence of cell wall stressors. When grown on plates with CW (20 μg/ml), SDS (0.005% [wt/vol]), CAS (0.025 μg/ml), or CR (50 μg/ml), tSEC6 plus DOX grew poorly on YNB agar supplemented with CW (Fig. 6). This was consistent with previous studies where strains with elevated chitin content were also found to be hypersensitive to CW (41). The tSEC6 strain plus DOX also grew poorly on CSM agar supplemented with SDS, which perturbs membrane integrity. Additionally, the tSEC6 strain plus DOX grew as well as control strains on agar plates with either CR or CAS (Fig. 6).

**FIG 6:** Growth of the tSEC6 strain under conditions of cell wall stress. Replicates of serial dilutions of cells were prepared on plates containing cell wall stressors (the four types of cells included in the experiment are listed at the top and correspond to the four rows for each stressor). The triangle at the bottom indicates decreasing cell densities (1.0 × 10^8^, 2.0 × 10^7^, 4.0 × 10^6^, 8.0 × 10^5^, 1.6 × 10^5^, and 3.2 × 10^4^ cells/ml, from left to right). There was no difference in growth between the strains grown on complete synthetic medium. Cell wall stressors were CAS, CR, CFW, and SDS. Under repressing conditions (+DOX), C. albicans tSEC6 grew poorly in the presence of CW and SDS.

To address the discrepancy in the results of these enzymatic assays, which indirectly assessed beta-glucan content, we next directly assayed cell wall composition in the tSEC6 and THE1-CIp10 strains by using HPAEC-PAD. These analyses revealed that glucan content was similar between the controls and tSEC6, but an increase in chitin content with a corresponding decrease in mannan content was observed in the mutant (Table 3). Although these differences were not statistically significant (*P* = 0.30), the overall trend was consistent with the sensitivity of the conditional tSEC6 mutant to CW (Fig. 6) and the increase of chitin staining by CW at the sites of cell division (Fig. 3A).

**TABLE 3:** Cell wall component analysis of Candida albicans strains

Strain (presence of DOX in medium)	Component % of cell wall^*a*^		
	Chitin	Glucan	Mannan
THE1-CIp10	3.42 ± 1.23	59.90 ± 3.37	36.67 ± 4.51
THE1-CIp10 (+DOX)	3.42 ± 1.23	60.19 ± 2.96	36.38 ± 4.06
tSEC6	4.33 ± 1.40	59.76 ± 2.68	37.63 ± 4.76
tSEC6 (+DOX)	8.22 ± 3.22	60.11 ± 3.22	31.68 ± 6.25

a Results represent the averages and standard deviations of five biological replicates.

RETRACTED

### Repression of *SEC6* results in defects in hypha formation.

One of the virulence traits implicated in C. albicans pathogenesis is the ability to switch between hyphal and yeast forms of growth (16). Thus, we examined the tSEC6 mutant under conditions that are optimal for hyphal growth on solid and in liquid media for up to 24 h. When incubated on agar medium, there was a clear impairment of filamentation in the tSEC6 mutant with DOX compared to the controls (Fig. 7).

**FIG 7:** Filamentation on solid hypha-inducing medium. Filamentation was analyzed using four different types of hypha-inducing medium: cells spotted on YPD with 10% (vol/vol) FCS, colonies embedded in YPD, and cells spotted on M199 or Spider medium. Images (10× magnification) are shown for YPD-embedded colonies and cells spotted on Spider and M199 media. A severe defect in filamentation was observed in the tSEC6 strain grown under restrictive conditions. Images were acquired after 24 h at 37°C; embedded cells in YPD agar were incubated at 30°C for 24 h.

We also tested *in vitro* filamentation in liquid, buffered RPMI. After inducing filamentation for 24 h, cultures of control cells were composed of approximately 20% yeast cells and 80% filamentous cells, whereas the proportion of tSEC6 plus DOX cells was 55% yeast cells and 45% filamentous cells (data not shown). Compared to control strains, a marked reduction in the number of branches in the hyphal cells in tSEC6 with DOX was observed (Fig. 8A). Quantification of the percentage of branched hyphae in those cells that were able to produce hyphae in all strains showed that the number of hyphal branches was significantly decreased in tSEC6 plus DOX (*P* < 0.05) (Fig. 8B). To ensure that these observations were not a direct result of arrest in growth of the tSEC6 strain under filamentation-inducing conditions, we assessed cell viability by enumerating CFU from each culture. The number of CFU in the tSEC6 plus DOX culture was similar to the CFU of the THE1-CIp10 plus DOX culture and derepressed THE1-CIp10 and tSEC6 cultures (*P* > 0.05) (data not shown), indicating that the defect in filamentation of the tSEC6 plus DOX cultures was not a result of decreased cell viability.

**FIG 8:** Assessment of the hyphal branching pattern of the tSEC6 strain. The number of lateral branches was quantified after 15 h of incubation in YPD (with or without DOX) and subsequent induction of filamentation in YPD with 20% (vol/vol) FCS for 8 h at 37°C with or without DOX. Experiments were performed in triplicate with 100 cells counted per treatment per experiment. (A) Light microscopy of the tSEC6 strain grown with or without DOX showed differences in branching patterns. Arrows indicate branches counted for each filament (4 total branches for the tSEC6 strain without DOX and 0 branches for the tSEC6 strain with DOX). Bar, 10 μm. (B) The proportion of hyphae with the indicated number of branches of each strain grown in the presence of absence of DOX. Strain tSEC6 grown with DOX had a decrease in the number of filaments with more than one branch. The asterisk indicates a statistically significant difference from the controls (*P* < 0.001).

RETRACTED

### *SEC6* expression is required for secretion of aspartyl proteases and lipases.

We next tested for defects in secretion of virulence-associated degradative enzymes, including Saps and lipases. In THE1-CIp10, complete proteolysis of extracellular BSA occurred (Fig. 9A), but BSA was not degraded by a mutant strain [*sap*Δ(1-3)] that does not express secreted aspartyl proteases Sap1, Sap2, and Sap3 (30). Strain tSEC6 with DOX was similarly unable to degrade BSA, indicating a defect in secretion of Saps. The tSEC6 mutant plus DOX also exhibited a substantial reduction in secreted lipase activity (Fig. 9B). These results indicated that *SEC6* plays an important role in the secretion of Saps, extracellular lipases, and presumably other secreted proteins.

**FIG 9:** Secretion of extracellular degradative enzymes by tSEC6 strain. (A) Cells from overnight cultures were transferred to BSA medium and incubated for 24 h to induce secretion of aspartyl proteases. The cells were then washed and concentrated into fresh BSA medium with or without DOX and incubated for 24 h with shaking. Supernatants collected from these cultures were analyzed by SDS-PAGE and subsequently stained with Coomassie blue to visualize the extent of BSA degradation that occurred as a result of proteolytic cleavage by Saps released into the medium. Liquid BSA medium alone was used as a control. The triple deletion mutant *sap*Δ(*1-3*) was also included as a negative control. Bands of intact BSA are indicative of reduced secretion of Saps. BSA degradation was markedly reduced in the tSEC6 strain grown with DOX compared to wild-type controls. (B) Secretion of degradative lipases was also assessed. Cells were grown overnight in liquid YPD and transferred to Tween 80 medium for 24 h to induce production and secretion of lipases. The cells were then washed and concentrated in fresh Tween 80 medium with or without DOX and incubated for 24 h at 37°C. The supernatant was collected and used in a turbidimetric kinetic assay that measured increases in optical density (500 nm) as a result of the precipitation of calcium salts formed when degradative products are combined with CaCl_2_. The rate of increase in the OD_500_ is proportional to the concentration of lipase present in the supernatant. Three biological replicates are represented and show a significant difference between the tSEC6 strain grown with DOX and the controls (*P* < 0.05). Error bars indicate standard deviations.

RETRACTED

### The *SEC6* mutant is defective in macrophage killing.

Phagocytes (macrophages) are one of the host's first lines of defense against Candida infection (42). Therefore, to assess virulence potential *in vitro*, we used a macrophage killing assay to analyze the effect of repression of *SEC6*. After coincubation of macrophages and C. albicans for 24 h, the control strains efficiently killed macrophages, as expected (Fig. 10A and B). In contrast, macrophage killing was reduced 3-fold when the cells were incubated with tSEC6 plus DOX, with a significant impairment compared to control strains (*P* < 0.05) (Fig. 10A and B).

**FIG 10:** tSEC6 shows impaired macrophage killing *in vitro*. (A) Following coincubation with C. albicans, macrophages were stained with calcein AM (live cells) and ethidium bromide homodimer (dead cells) and visualized by fluorescence microscopy. Representative images from three independent experiments, incubated for 24 h, are shown. The right lower panel shows an increase in live macrophages, which is indicative of defective macrophage killing by the tSEC6 mutant strain. (B) The average numbers of live macrophage cells from 12 separate fields after 24 h of coincubation with C. albicans strains are shown. Error bars indicate standard deviations. The asterisk indicates a statistically significant difference (*P* < 0.05) between tSEC6 in the presence of DOX versus control strains.

## DISCUSSION

The exocyst complex has been extensively studied in S. cerevisiae (43, 44) and is required for polarized exocytosis in multiple organisms, including C. albicans, where secretion is vital for growth of yeast and hyphal cells, and the delivery of secreted enzymes influences pathogenesis and the host-pathogen interaction. To expand our understanding of the function of the C. albicans exocyst, we performed a detailed investigation of each component of the complex and have presented here our findings for C. albicans SEC6. In S. cerevisiae, *SEC6* encodes an 85-kDa protein composed of 733 amino acids; it is predicted to be hydrophilic, and it is found in the soluble fraction of the yeast lysate (45). Using the National Center for Biotechnology Information (NCBI) protein Basic Local Alignment Search tool (BLASTp [46]) and the Candida Genome Database (CGD [47]), we identified a homologous predicted protein in C. albicans (orf19.5463) that has 24% identity and 45% similarity with S. cerevisiae Sec6. Because *SEC6* is essential in S. cerevisiae, we constructed a conditional mutant to analyze gene function in C. albicans. Growth assays indicated that *SEC6* is also essential for viability in C. albicans, with cell death occurring 27 h after *SEC6* expression was repressed. Additionally, the C. albicans tSEC6 conditional mutant exhibited striking morphological defects in both the yeast and hyphal forms. The majority of tSEC6 yeast cells were round instead of exhibiting a typical ellipsoidal shape, and their size was enlarged. We also found marked accumulation of secretory vesicles in the conditional mutant, a phenotype that has been observed in S. cerevisiae temperature-sensitive mutants (e.g., S. cerevisiae sec6-4). Intracellular accumulation of vesicles has been associated with defects in secretion (3, 5), and it is likely that these accumulated vesicles are associated with decreased secretion of extracellular proteases and lipases in the C. albicans tSEC6 conditional mutant.

RETRACTED

Septins have a well-established role in cytokinesis and septum formation. Septins are filamentous GTP-binding proteins that have been implicated in fungi in multiple processes, including cell separation, conjugation, sporulation, and recruitment of proteins to the bud neck (48–50). In both C. albicans and S. cerevisiae, four septins (Cdc3, Cdc10, Cdc11, and Cdc12) have been described to form a ring on the inner surface of the plasma membrane at the bud neck during cell division (50). The process of cell division can be classified into two steps in terms of septin ring formation: (i) formation of a septin hourglass structure that is observed between the anaphase and telophase stages of the cell division cycle, and (ii) formation of a two-ring structure before the onset of cytokinesis, resulting from splitting of the major ring. It has been proposed that the exocyst mainly functions in the second step (septin double rings), where vesicle trafficking increases due to a rise in demand for cell wall remodeling components, including cell wall hydrolases and glucan synthases (50, 51). We found an elongated septin ring at the bud neck in the conditional mutant compared to the control strains. Moreover, the defect in cell division in the tSEC6 mutant strain was accompanied by a localized increase in chitin content at the site of the septum. Based on previous observations in S. cerevisiae (48), it is likely that the supply of proteins necessary for mother and daughter cells to separate is interrupted in the absence of Sec6. Our results suggest that septum morphology is altered in the conditional mutant; interestingly, a previous study showed that septin mutants of C. albicans (particularly the *cdc10*Δ null mutant) displayed defects in cytokinesis, diffuse mislocalization of chitin, and increased axial bud scars (35). The conditional tSEC6 strain also displayed defects in cytokinesis and a high degree of axial budding, but in contrast to the *cdc10*Δ null mutant, we observed a focal increase in chitin content at the bud neck.

RETRACTED

Repression of *SEC6* also resulted in hypersensitivity to the cell wall stressors CW and SDS. Zymolyase, CR, and CAS affect cell wall composition by inhibiting the synthesis of β-1,3-glucan (52, 53), whereas chitinase degrades chitin in the cell wall. CW binds to nascent chitin and represses its deposition in chains, resulting in inhibition of growth (54). In agreement with previous studies where it has been shown that a decrease in content of one of the main C. albicans cell wall components (glucan, chitin, and mannoproteins) results in a compensatory effect in order to maintain cell wall integrity (52, 55, 56), we observed a trend toward decreased mannose and increased chitin content in the tSEC6 mutant strain cultured with DOX, although these differences were not statistically significant. The observed increased resistance to chitinase degradation was consistent with the raised levels of chitin in the cell wall of the tSEC6 strain grown under repressing conditions. However, it was interesting to also see increased resistance to zymolyase degradation despite the unaltered total glucan content. The resistance to zymolyase could be a result of structural changes in the glucan network in the tSEC6 mutant strain. One possibility is that repression of *SEC6* results in trafficking defects which impair delivery of cell wall maintenance and remodeling enzymes. Alternatively, there may be alterations in cell wall structure in the conditional mutant that cause architectural changes in the cell wall, making it less accessible to degradation by zymolyase and chitinase.

Under repressing conditions, the tSEC6 mutant had a striking impairment in filamentation, producing hyphae that lacked the normal branching pattern. During hyphal development of wild-type strains, true hyphae grow with parallel cell walls (57). In the conditional mutant, hyphal cells were less parallel in the distal segments and, notably, exhibited a marked decrease in formation of lateral branches. We also studied the contribution of Sec6 to pathogenesis by performing an *in vitro* model of macrophage infection (34). Macrophage killing was significantly attenuated in the conditional mutant grown under repressing conditions compared to the controls. Wild-type C. albicans strains induce macrophage death by forming filaments in response to the phagosome environment (34, 58). Thus, it is likely that the severe defect in filamentation was responsible for the attenuated virulence in macrophages. Taken together, we have demonstrated that C. albicans *SEC6* is required for polarized growth, which is vital for tissue penetration, lateral branching of hyphae, cytokinesis, and the secretion of virulence-associated enzymes.

RETRACTED

Our recent work on C. albicans t-SNAREs Sso2 and Sec9 demonstrated their role in hyphal growth and secretion; however, the conditional mutants exhibited clear phenotypic differences despite their predicted interactions in the SNARE complex (3). Repression of *SSO2*, but not *SEC9*, resulted in hyphal growth arrest and a return to isotropic growth with a corresponding loss of the C. albicans Spitzenkörper at the hyphal tip. Interestingly, when grown under hypha-inducing conditions as described previously (3), the Spitzenkörper is also still present at the hyphal tip of the tSEC6 strain when grown under repressing conditions (A. A. Chavez-Dozal et al., unpublished results). This similarity can be explained in part by the suggested physical interaction of Sec6 and Sec9 in S. cerevisiae (8), which brings two proteins from different complexes together, spatially and temporally, in a key step in exocytosis. It is further believed that release of Sec9 from this interaction allows formation of the SNARE complex (8) and is concomitant with binding of Sec6 with other components of the exocyst complex (10), leading to fusion between the vesicles and target membranes. As we continue our detailed examination of the role of the individual subunits of the exocyst in C. albicans, we are finding differences in their involvement in secretion and polarized growth that are distinct from those reported in previously published work regarding S. cerevisiae and that represent a novel finding in this opportunistic pathogen. It would be of further interest to see if these findings extend to filamentous fungi and/or are limited to pathogenic fungi.

## Supplementary Material

Supplemental material
